# Gastroprotective Effect of Myricetin on Ethanol-Induced Acute Gastric Injury in Rats

**DOI:** 10.1155/2021/9968112

**Published:** 2021-09-29

**Authors:** Hee-seon Park, Chang-Seob Seo, Eun Bok Baek, Jin-hyung Rho, Young-Suk Won, Hyo-jung Kwun

**Affiliations:** ^1^Department of Veterinary Pathology, College of Veterinary Medicine, Chungnam National University, Daejeon 34134, Republic of Korea; ^2^Herbal Medicine Research Division, Korea Institute of Oriental Medicine, Daejeon 34054, Republic of Korea; ^3^Laboratory Animal Resource Center, Korea Research Institute of Bioscience and Biotechnology, Cheongju, Republic of Korea

## Abstract

The flavonoid myricetin is abundant in vegetables and has various bioactive properties, including anti-inflammatory and antioxidative activities. In the present study, we explored the effects of myricetin on alcohol-induced gastric ulcer in a rat model. To induce gastric ulcer, absolute ethanol (5 mL/kg body weight) was orally administrated to each rat. The positive control and myricetin-treated groups were given oral doses of omeprazole (20 mg/kg) or myricetin (12 mg/kg), respectively, 1 hour prior to the administration of absolute alcohol. We found that pretreatment with myricetin significantly decreased alcohol-induced gastric ulcer, hemorrhage, hyperemia, and epithelial cell loss in the gastric mucosa. Myricetin pretreatment reduced the level of malondialdehyde (MDA) and increased that of total glutathione (GSSG/GSH) and superoxide dismutase (SOD) in gastric tissues. In addition, it elevated the expression levels of cyclooxygenase-1 (COX-1) and prostaglandin E_2_ (PGE_2_) and decreased the phosphorylation of nuclear factor kappa B (NF-*κ*B). Together, these results indicate that myricetin effectively inhibits ethanol-induced acute gastric injury by preventing oxidative damage, stimulating PGE_2_ production, and inhibiting NF-*κ*B activation. We suggest that myricetin may be an alternative treatment for gastric injury caused by alcohol intake.

## 1. Introduction

Gastric ulcer (also known as peptic ulcer) is a major gastrointestinal disorder whose global incidence and prevalence are on the rise. The prevalence of gastric ulcer is estimated at 0.2–0.5% in Western countries and 2-3% in Asian countries, and recurrence rates are as high as 60% [1]. The lesion has multiple etiologies associated with perturbation of the balance between factors that seek to protect or damage the mucosal epithelium [2]. The damaging factors can include overuse of nonsteroidal anti-inflammatory drugs (NSAIDs), smoking, *Helicobacter pylori* (*H. pylori*) infection, alcohol consumption, and psychological and physiological stress [3]. Among them, excessive alcohol drinking is considered to be the leading cause of gastric mucosal damage [4].

The strategies currently used to treat gastric ulcer are based on the cause of the ulcer; they include the use of proton-pump inhibitors, antibiotics aimed at eradicating *H. pylori* infection (if present), and the application of histamine type-2 receptor blockers that reduce acid production [5]. Stomach acid-neutralizing antacids and cytoprotective agents, such as sucralfate and misoprostol, may also be employed. However, many of these drugs can have undesirable adverse effects and impose a cost burden on gastric ulcer patients [6, 7]. Therefore, researchers continue to seek new agents that can be used to treat gastric ulcer with greater safety, fewer side effects, higher efficiency, and lower cost.

Myricetin (3,5,7-trihydroxy-2-(3,4,5-trihydroxyphenyl)chromen-4-one) is a natural flavonoid that belongs to the flavonol subclass and is commonly found in vegetables, fruits, berries, medicinal herbs, and tea [8]. It is particularly notable in certain natural products, including fresh broad beans (*Phaseolus vulgaris*), black tea, broccoli (*Brassica oleracea*), bell pepper (*Capsicum annuum*), and garlic (*Allium sativum*) [9]. Myricetin has multiple biological properties, including antioxidant [10], antimicrobial [11], antiviral [12], anti-inflammatory [13], antitumor [14], analgesic [15], hepatoprotective [16], hypoglycemic [17], hypolipidemic [18], cardioprotective [19], and neurological damage-inhibiting [20] actions. Myricetin suppresses gastric H^+^, K^+^-ATPase in the gastrointestinal tract and thus could be a useful starting compound for developing new agents to alleviate gastric acid secretion [21]. In addition, myricetin has been shown to prevent ulcerative colitis and colorectal tumor in dextran sulfate sodium- (DSS-) induced model mice [22, 23]. Based on the previous reports, we hypothesized that myricetin may have antiulcerogenic potential in the stomach. Here, we investigated the protective effect of myricetin in a rat model of ethanol-induced gastric injury.

## 2. Materials and Methods

### 2.1. Chemical

We obtained myricetin (CAS No. 529-44-2; purity, 97.8%) from Tokyo Chemical Industry Co., Ltd. (Tokyo, Japan).

### 2.2. Animals

Male 6- to 7-week-old Sprague Dawley (SD) rats weighing 150–250 g were provided by Orient Bio (Republic of Korea). Animals were raised in a constant temperature (23 ± 2°C) with a regular 12 : 12-h light : dark cycle and acclimated for 1 week prior to experiments, as previously described [2, 24, 25]. Animal experiments were approved by the Animal Experimental Ethics Committee of Chungnam National University (approval number: CNU-00444) and were performed in compliance with the National Institutes of Health Guide for the Care and Use of Laboratory Animals.

### 2.3. Experimental Design

Gastric lesions were induced by oral administration of absolute ethanol, as previously described [2, 24, 25]. Rats were randomly divided into the following four groups (Table 1; *n* = 6-7 per group): normal control (NC), ethanol (EtOH), omeprazole + EtOH (Ome + EtOH), and myricetin + EtOH (Myr + EtOH). Animals were fasted for 24 h prior to induction. Rats of the NC group were given 5 mL/kg body weight (b.w.) phosphate-buffered saline (PBS; vehicle), while those in the EtOH, Ome + EtOH, and Myr + EtOH groups were given the same volume (5 mL/kg b.w.) of absolute ethanol by oral gavage. At 1 h prior to alcohol administration, the Ome + EtOH group was given an oral dose of omeprazole (20 mg/kg b.w.) and the Myr + EtOH group was given myricetin (12 mg/kg b.w.). The dose of myricetin was determined according to a previous dosing experiment of ethanol-induced ulceration on rats. At 1 h after ethanol treatment, all animals were sacrificed by overdoses of 50 mg/kg pentobarbital, and stomachs were collected.

### 2.4. Macroscopic Determination of Gastric Ulcer Area

Stomachs were collected and dissected along the greater curvature, and the gastric mucosa was rinsed with normal saline. Stomach tissues were flattened and photographed. Image analysis software (ImageJ 46a; NIH, USA) was used to analyze the ulcerated area (UA; mm^2^), and the ratio of UA to gastric area and the inhibition percentage were analyzed. The inhibition percentage was calculated as follows: ((UA control − UA treated)/UA control)) × 100%.

### 2.5. Histopathological Examination

Stomach tissues were fixed in 10% neutral buffered formalin (NBF), paraffin-embedded by routine histopathological methods, sectioned at 4 *µ*m, and stained with hematoxylin and eosin (H&E).

### 2.6. Determination of Malondialdehyde (MDA), Total Glutathione (GSSG/GSH), and Superoxide Dismutase (SOD)

To analyze MDA, stomach samples were prepared in PBS with butylated hydroxytoluene (BHT) to prevent further oxidation. The tissue homogenates were centrifuged at 10,000 g for 5 min, supernatants were collected, and MDA levels were determined using a commercially available kit (Cell Biolabs, USA). The levels were normalized based on the total protein concentration of each lysate. For assessment of total glutathione, tissue lysates were prepared in 5% metaphosphoric acid (MPA) and centrifuged at 12,000 rpm for 15 min at 4°C, and total glutathione was assessed using a commercially available kit (Cell Biolabs) and normalized by the protein concentration. For activity assessment of the antioxidative enzyme, SOD, stomach tissues were homogenized in PBS and centrifuged, and collected supernatants were assessed for SOD activity using a commercially available kit (Cayman, USA). The results were normalized by the protein concentration and are expressed as U/mg protein. The protein concentrations used for normalization were determined by the Bradford method.

### 2.7. Determination of Prostaglandin E_2_ (PGE_2_)

Stomach tissue samples were homogenized and centrifuged, and supernatants were assessed for PGE_2_ using a commercially available kit (Cayman, USA). Absorbance was measured at 450 nm with an ELISA microplate reader (Bio-Rad Laboratories, USA).

### 2.8. Western Blot Analysis

Stomach tissues were dissected and ground in radioimmunoprecipitation assay (RIPA) buffer (Cell Signaling Technology, USA) containing phosphatase and protease inhibitors (Roche, Germany). The samples were centrifuged, and supernatants were collected. The protein content was analyzed by the Bradford method. Tissue proteins were separated by 8% sodium dodecyl sulfate-polyacrylamide gel electrophoresis (SDS-PAGE), transferred to a polyvinylidene fluoride (PVDF) membrane (Millipore, USA) at 350 mA for 2 h, blocked by incubation with 5% bovine serum albumin (BSA) in PBS containing 0.1% Tween 20 (PBS-T) for 1 h, and then incubated overnight with primary antibodies at 4°C. The utilized antibodies recognized phospho-nuclear factor kappa B (p-NF-*κ*B), NF-*κ*B (Cell Signaling Technology), and *β*-actin (Sigma-Aldrich, USA). After being washed with PBS-T, membranes were exposed to rabbit or mouse secondary antibodies, as appropriate, for 2 h and developed using a western blot chemiluminescent substrate (Thermo Scientific, USA).

### 2.9. RNA Isolation and Quantitative Real-Time PCR Analysis

RNA was isolated with TRIzol reagent (Invitrogen, USA) in accordance with the manufacturer's protocol. The level of RNA was assessed by the intensity at 260 nm, and its purity was determined based on the intensity ratio of 260 nm to 280 nm. RNA was reverse transcribed (ReverTra Ace kit, Toyobo, Japan), and the expression levels of the mRNAs of interest were measured using a StepOnePlus Real-Time PCR System (Applied Biosystems, USA). The relative transcript level was calculated from duplicate samples after the results were normalized by the mRNA expression of glyceraldehyde-3-phosphate dehydrogenase (GAPDH). The utilized primer pairs and PCR condition are listed in Table 2. PCR data ware expressed as the fold change of the target gene relative to the level of GAPDH, as calculated using the 2^-ΔΔ*Ct*^ method.

### 2.10. Statistical Analysis

Data are expressed as means ± standard deviation (SD). Statistical significance was determined using one-way analysis of variance (ANOVA), and the significance between the groups was analyzed by Tukey's multiple comparison test. *P* values <0.05 were considered significant.

## 3. Results

### 3.1. Effect of Myricetin on Ethanol-Induced Acute Gastric Injury

No injury was found in the normal control group (Figure 1(a)). Severe ulcers accompanied by elongated-band hemorrhage were detected in the glandular layer of the stomach in rats from the ethanol-administered group (Figure 1(b)), but this ethanol-induced gastric injury was attenuated in the omeprazole- and myricetin-pretreated groups (Figures 1(c) and 1(d)). The UA in the alcohol-treated group was 174.3 ± 41.7 mm^2^, whereas that in rats pretreated with omeprazole or myricetin was 54.0 ± 42.8 mm^2^ (69% inhibition) and 74.2 ± 19.1 mm^2^ (57% inhibition), respectively (Table 3). Histopathological analyses showed severe hemorrhage, extensive submucosal edema, and the loss of gastric mucosa from stomach tissues of ethanol-treated rats (Figure 2(b)), but this ethanol-induced damage was notably reduced by omeprazole or myricetin pretreatment (Figures 2(c) and 2(d)). These results indicate that myricetin significantly decreased alcohol-induced gastric ulcer and injury in the rat model.

### 3.2. Effect of Myricetin on Lipid Peroxidation and Antioxidant Enzymes

The MDA level in stomach tissue was markedly enhanced in ethanol-treated rats compared to the normal control group. Omeprazole or myricetin pretreatment significantly decreased this ethanol-induced increase in MDA (Figure 3(a)). The gastric total glutathione concentration and SOD activity were lower in the ethanol-treated group than in the normal control group, but omeprazole or myricetin pretreatment significantly attenuated these decreases, such that the total glutathione concentration and SOD activity were higher in the omeprazole- and myricetin-pretreated groups than the ethanol-treated group (Figures 3(b) and 3(c)). These findings suggest that myricetin significantly alleviated the oxidative stress induced by ethanol administration.

### 3.3. Effect of Myricetin on Activation of NF-*κ*B

Western blot analyses showed that phosphorylation of NF-*κ*B in stomach tissues was increased in the ethanol-treated group compared with the normal control group, but omeprazole or myricetin pretreatment significantly attenuated NF-*κ*B activity compared with the ethanol-treated group (Figure 4). This indicates that myricetin exerts protective activity through suppression of the NF-*κ*B-dependent pathway.

### 3.4. Effect of Myricetin on the Expression of Cyclooxygenase-1 (COX-1) and PGE_2_

The mRNA expression level of COX-1 was elevated after ethanol administration, and this increase was significantly enhanced by pretreatment with omeprazole or myricetin (Figure 5(a)). The level of PGE_2_ was slightly lower in rats subjected to intragastric administration of ethanol compared with the normal control group, but this level was significantly increased by pretreatment with omeprazole or myricetin (Figure 5(b)). These results suggest that myricetin might show protective effects on ethanol-induced gastric injury at least partially via COX-1 and PGE_2_.

## 4. Discussion

Myricetin is a flavonoid that offers numerous pharmacological benefits, such as antioxidant, anti-inflammatory, and anticancer activities [10, 13]. Here, we assessed the potential pharmacologic effects of myricetin against ethanol-induced gastric mucosal injury in SD rats. We found that myricetin pretreatment protected gastric tissue against acute injury induced by absolute alcohol, suppressing gastric injury, lipid peroxidation, and NF-*κ*B activation while increasing antioxidant activity and PGE_2_ expression.

Ethanol-induced stomach ulceration is a classic model that is often used in studies assessing the protective effects of drugs in the stomach, particularly cytoprotective and/or antioxidant activities [26, 27]. Upon administration, ethanol rapidly penetrates the gastric mucosa; this exposes the mucosal layer to hydrochloric acid and pepsin [28], which have proteolytic and hydrolytic effects that damage cell membranes to cause cell exfoliation, erosion, and ulcer [29]. Here, we show that myricetin pretreatment inhibited ulceration by ∼57% in this model and thus showed an efficacy similar to that of omeprazole. The antiulcer effect of myricetin was supported by our histopathological examination, which revealed that myricetin-administered rats had intact mucosal structures and glandular elements, along with decreases in submucosal edema and hemorrhage. These results indicate that myricetin protects the stomach against ethanol-induced injury to the gastric mucosa.

Gastric lesions induced by alcohol are closely related to the generation of reactive oxygen species (ROS), reflecting that lesions are associated with an imbalance between oxidative and antioxidative cellular processes [30]. This shift to an oxidative state arises from the release of hydroperoxy free radicals and superoxide anions, whose increases cause an oxidative stress that can be visualized as an increased level of MDA [31, 32]. MDA is generated by the peroxidation of polyunsaturated fatty acids or related esters within cell membranes and is used as a marker of ROS-induced cellular damage [33]. GSH and SOD are among the defense mechanisms that protect cells against ROS-induced lipid peroxidation [34]. GSH inhibits lipid peroxidation and scavenges radicals; it is among the most abundant cellular antioxidants and acts to detoxify hydrogen peroxide by various glutathione peroxidases [35]. SOD, meanwhile, acts on superoxide produced during oxidative stress, converting it to hydrogen peroxide [36]. In the present study, oral administration of alcohol markedly increased the levels of MDA and decreased those of total glutathione and SOD activity, supporting the notion that oxidative stress plays an important role in the pathogenesis of ethanol-induced gastric injury. Pretreatment with myricetin markedly increased the level of SOD and total glutathione and decreased that of MDA. These findings are consistent with previous reports that myricetin exerts a strong antioxidant activity by scavenging hydroxyl free radicals [37] and can restore cellular antioxidant defense enzymes, including SOD, catalase (CAT), and glutathione peroxidase (GPx) [38]. Taken together, our results indicate that myricetin appears to exert a gastroprotective effect via an antioxidant mechanism.

ROS activates NF-*κ*B, which is a critical regulator that promotes the transcription of genes related to inflammation, cell survival, and immune responses. During ethanol-induced gastric ulcer formation, NF-*κ*B governs the increased transcription of genes encoding inducible nitric oxide synthase (iNOS), COX-2, and inflammatory cytokines including tumor necrosis factor-*α* (TNF-*α*), interleukin (IL)-6, and IL-1*β* [2]. NF-*κ*B expression is therefore a crucial nexus for gastric ulcer formation, making it a logical target for the treatment of inflammatory conditions [39]. Here, we found that alcohol administration induced a remarkable increase of NF-*κ*B that was significantly suppressed by pretreatment with myricetin. These results are consistent with previous reports that myricetin exerts anti-inflammatory activity by suppressing I*κ*B kinase/NF-*κ*B-dependent signaling [40,41].

Gastric mucosal cells produce prostaglandins (PGs), which function as important endogenous mediators during acute gastric mucosal injury [42,43] and contribute to mucosal defense by regulating the secretion of acid and stimulating those of mucus, bicarbonate, and phospholipids. PGs also accelerate epithelial restitution and mucosal healing [44] and mediate inflammatory reactions by increasing vascular permeability, leading to vasodilation and increased blood flow [45]. PGs are generated by COX enzymes; among them, COX-1 produces PGs that play essential roles in homeostatic functions, including maintenance of mucosal integrity and mucosal blood flow [46]. Here, we found that the levels of COX-1 and PGE_2_ (the most abundant prostaglandin [47]) were significantly higher in the myricetin-pretreated group than in the alcohol-treated group. This suggests that myricetin acts via COX-1 and PGE_2_ to exert protective effects against ethanol-induced gastric mucosal injury.

We herein used omeprazole, a proton-pump inhibitor that suppresses gastric acid secretion [5], as a positive control. As omeprazole can produce undesirable adverse effects and impose a cost burden on gastric ulcer patient [6, 7], there is increasing demand for alternative strategies that can treat gastrointestinal diseases with fewer adverse effects. Myricetin was previously shown to inhibit H^+^, K^+^-ATPase and attenuate gastric acid secretion, suggesting its potential to alleviate gastric acid-related diseases when used alone or in a combination treatment [21]. The present study demonstrates the first evidence that myricetin may have gastroprotective effects against alcohol-induced gastric ulcer. The gastroprotective effects of myricetin appear to be at least partially mediated by its ability to reduce oxidative stress, inhibit NF-*κ*B, and stimulate PGE_2_ secretion. Further studies are needed to confirm that myricetin is a viable alternative for the clinical management of gastric ulcer diseases.

## 5. Conclusion

Our study results indicate that myricetin effectively inhibits ethanol-induced acute gastric injury by preventing oxidative damage, stimulating PGE_2_ production, and inhibiting NF-*κ*B activation. Myricetin may be an alternative treatment for gastric injury caused by alcohol intake.

## Figures and Tables

**Figure 1:** Gross findings of the gastric mucosa. (a) Normal control group. (b) Ethanol-treated group. (c) Omeprazole plus ethanol-treated group. (d) Myricetin plus ethanol-treated group.

**Figure 2:** Histopathological examination of gastric tissue. (a) Normal control group. (b) Ethanol-treated group. (c) Omeprazole plus ethanol-treated group. (d) Myricetin plus ethanol-treated group. No disturbance in the gastric mucosa was detected in the normal control group, whereas the ethanol-treated group showed severe destruction of the surface epithelium and necrotic lesions. The black arrow indicates severe hemorrhage of the mucosal layer. Magnification, ×100 and ×400.

**Figure 3:** Levels of MDA, total glutathione (GSSG/GSH), and SOD in stomach tissue. (a) MDA concentration. (b) Total glutathione concentration. (c) SOD activity. Values represent means ± SD (^#^*P* < 0.05 and ^##^*P* < 0.01 compared to the normal control group; ^*∗*^*P* < 0.05 and ^∗∗^*P* < 0.01 compared to the ethanol-treated group).

**Figure 4:** NF-*κ*B activity. Values represent means ± SD (^#^*P* < 0.05 and ^##^*P* < 0.01 compared to the normal control group; ^*∗*^*P* < 0.05 and ^∗∗^*P* < 0.01 compared to the ethanol-treated group).

**Figure 5:** Expression of COX-1 and production of PGE_2_. (a) COX-1 mRNA levels. (b) PGE_2_ levels. Values represent means ± SD (^#^*P* < 0.05 and ^##^*P* < 0.01 compared to the normal control group; ^*∗*^*P* < 0.05 and ^∗∗^*P* < 0.01 compared to the ethanol-treated group).

**Table 1:** Animal study group design.

Group	Treatment (dose)
NC	PBS (5 mL/kg body weight) + PBS (5 mL/kg body weight)
EtOH	PBS (5 mL/kg body weight) + ethanol (5 mL/kg body weight)
Ome + EtOH	Omeprazole (20 mg/kg body weight) + ethanol (5 mL/kg body weight)
Myr + EtOH	Myricetin (20 mg/kg body weight) + ethanol (5 mL/kg body weight)

**Table 2:** Primer pairs used for qRT-PCR.

*Primer sequence*			
Cox-1	F: 5′-TGACTATCTGGCGGGTGACT-3′ R: 5′-CTTGCTGGACATTGGGTTCT-3′		
Gapdh	F: 5′-ACAGCAACAGGGTGGTGGAC-3′ R: 5′-TTTGAGGGTGCAGCGAACTT-3′		

*Real-time PCR condition*			
Step	Temperature (°C)	Time	Cycle
Initial denaturation	95	10 min	1
Denaturation	95	15 sec	40
Annealing and Extension	60	1 min	
Melt curve stage	95	15 sec	1
	60	1 min	

**Table 3:** Effects of myricetin on gastric ulcer area (UA, mm^2^) and percentage inhibition.

Group	Treatment	UA (mm^2^)	Inhibition (%)
NC	PBS + PBS	0.0 ± 0.0	—
EtOH	PBS + ethanol	174.3 ± 41.7^##^	—
Ome + EtOH	Omeprazole + ethanol	54.0 ± 42.8^∗∗^	69
Myr + EtOH	Myricetin + ethanol	74.2 ± 19.1^∗∗^	57

The results are expressed as mean ± SD. ^##^*P* < 0.01 compared to the NC group. ^∗∗^*P* < 0.01 compared to the EtOH group.

## Data Availability

The data generated from the findings of this study are included within the article.
